The article "Evaluating the relative contributions of copying and reconstruction processes in cultural transmission episodes" was published in 2021. Journal: PLoS One.

# Evaluating the relative contributions of copying and reconstruction processes in cultural transmission episodes

**DOI:** 10.1371/journal.pone.0256901

**Published:** 2021-09-16

**Authors:** James W. A. Strachan, Arianna Curioni, Merryn D. Constable, Günther Knoblich, Mathieu Charbonneau

**Affiliations:** 1 Cognition, Motion and Neuroscience Unit, Fondazione Istituto Italiano di Tecnologia, Genoa, Italy; 2 Department of Cognitive Science, Central European University, Vienna, Austria; 3 Northumbria University, Newcastle upon Tyne, United Kingdom; University of Queensland, AUSTRALIA

## Abstract

The ability to transmit information between individuals through social learning is a foundational component of cultural evolution. However, how this transmission occurs is still debated. On the one hand, the copying account draws parallels with biological mechanisms for genetic inheritance, arguing that learners copy what they observe and novel variations occur through random copying errors. On the other hand, the reconstruction account claims that, rather than directly copying behaviour, learners reconstruct the information that they believe to be most relevant on the basis of pragmatic inference, environmental and contextual cues. Distinguishing these two accounts empirically is difficult based on data from typical transmission chain studies because the predictions they generate frequently overlap. In this study we present a methodological approach that generates different predictions of these accounts by manipulating the task context between model and learner in a transmission episode. We then report an empirical proof-of-concept that applies this approach. The results show that, when a model introduces context-dependent embedded signals to their actions that are not intended to be transmitted, it is possible to empirically distinguish between competing predictions made by these two accounts. Our approach can therefore serve to understand the underlying cognitive mechanisms at play in cultural transmission and can make important contributions to the debate between preservative and reconstructive schools of thought.

## Introduction

Social learning, the mechanism of transmitting skills, ideas, and actions from one individual to another, plays a key role in stabilizing cultural traditions from one generation to the next [1]. The process by which it does so, however, is hotly debated within the field of cultural evolution [2–7]. One position is that social learning is mostly a copying process akin to mechanisms of genetic inheritance where social learners faithfully replicate the information required to learn and produce some behaviour and that cultural stability is a result of the preservation of this information [8–11]. Another position is that social learning depends on a process of reconstruction: Social learners reconstruct the information they believe to be the most relevant on the basis of pragmatic inferences, contextual information, and other constructive processes [6,12,13]. In the latter case, cultural stability arises because social learners tend to share the same constructive processes and common background knowledge.

The article "Evaluating the relative contributions of copying and reconstruction processes in cultural transmission episodes" was published in 2021. Journal: PLoS One.

Experimentally distinguishing between these two processes has been difficult since both copying and reconstruction can account for stable chains of cultural transmission [3,14,15]. If a learner’s output is similar to the input that they observed this may be interpreted as evidence of copying, but a reconstruction process can also explain input-output form similarities in stable transmission chains if the context leads learners to reconstruct the to-be-learned behaviour in the same way as the model [4,7,16]. There have been recent calls for empirical work to help settle this debate [2].

A key challenge to resolving this debate is thus to construct experimental settings that can differentiate between copying and reconstruction in interpersonal transmission. In this paper, we present a novel methodological approach that can empirically distinguish between copying and reconstruction, drawing on literature from cognitive psychology on joint action and coordination [17]. We start by describing the two competing accounts of social learning. We then present our methodological approach and explain how this generates competing predictions from the two accounts. Finally, we present the results of an experimental proof of concept that validates this novel approach.

## Two sides of the debate: Copying and reconstruction

In the cultural evolution literature, there is an ongoing debate as to how social learners successfully reproduce essential action features. In particular, the debate concerns what kinds of social learning mechanisms are primarily responsible for the apparently uniquely human capacity to transmit cultural items, and how these mechanisms contribute to the flexibility and stability of cultural traditions. Two candidate processes proposed by the different sides of this debate as being central to the human capacity to socially learn cultural information can be described as *copying* (sometimes referred to as preservation) and *reconstruction* [2–4,12]. The two accounts differ in terms of how they prioritise these mechanisms in terms of their importance for explaining the process of cultural transmission.

The copying account draws on the early emergence of the field of cultural evolution as inspired by the Darwinian theory of biological evolution, and this is strongly reflected in its emphasis on the faithful transmission of cultural traits [10,11,18]. According to this account, cultural transmission can be taken to follow a strict copying process where a learner observes a model produce a behaviour and copies it faithfully, replicating the behaviour in a ‘Xerox’ fashion. The high fidelity of copying is argued to be responsible for maintaining stable cultural traditions. Furthermore, exposure to complex inputs (such as observing many people with idiosyncratic ways of performing a technique) can result in blending or recombination of signals [19–21].

The article "Evaluating the relative contributions of copying and reconstruction processes in cultural transmission episodes" was published in 2021. Journal: PLoS One.

In a perfectly successful transmission episode, the copying account predicts that any output of a learner would be the result of information already present in the input signal (i.e. given the opportunity to observe a series of behaviour productions *A*, *B*, and *C* and their outcomes, the learner’s output product will be a copy of *A*, *B*, *C*, or some weighted combination thereof, but not *D*). Real-world transmission is never perfect, however—learners and the models they copy are noisy organisms embedded within noisy environments, and differences in body morphology and ecological affordances can introduce unavoidable variance into copied behaviours.

The copying account compensates for this noisiness by assuming a degree of random variation in learned behaviour, or copying errors [10]. That is, anything entirely new in the learner’s output that was not already present in the input (i.e. anything that cannot be determined by knowing *A*, *B*, or *C*), is the result of random copying error—the unavoidable consequence of a stochastic learning environment and imperfect cognition (e.g. faulty perception or memory, or poor motor skills). This high-fidelity replication is argued to be the driving force of stability in cultural traditions, while innovations and changes across generations are the result of accumulated random copying errors.

While cultural transmission can be considered a highly faithful copying process analogous to genetic inheritance [9,10,22], the cultural evolution literature typically approaches the idea with much more nuance than this analogy implies. The copying account proposes high-fidelity imitation as a prototypical preservative learning process. However, imitation is not ‘blind’ copying as with genetic inheritance. Rather, research in cognitive and developmental psychology shows that, when imitating, learners select which features of a behaviour they learn [23,24]. Further, imitation is often context-sensitive [25,26], and it operates at multiple degrees of abstraction [27].

The article "Evaluating the relative contributions of copying and reconstruction processes in cultural transmission episodes" was published in 2021. Journal: PLoS One.

For example, take a novice tennis player trying to learn how to serve a ball by watching his coach produce the action. As the coach prepares to show him the serve, she pauses and adjusts her hat to keep the sun from her eyes. If cultural transmission were truly analogous to genetic transmission, the learner would also pause to adjust his hat before he reproduces the behaviour even if it has suddenly become cloudy, as he copies everything that he has seen. Instead, the learner can understand that certain features of the observed behaviour (the actions of preparing and serving the ball) are *integral* to the to-be-learned information, while other features (such as adjusting one’s hat) are *incidental* and not supposed to be learned. Copying these incidental features would be over-imitation, as a learner misidentifies non-integral features as integral and so incorporates them into their action representation [28,29]. Differences between a model and a learner’s productions that appear only on incidental features are therefore not relevant to cultural transmission, while differences on integral dimensions of a behaviour are driven by random copying errors [30]. Moreover, the copying account does not deny the existence of other reconstructive learning mechanisms (just as the reconstruction account, below, does not deny the existence of copying), but argues that, of the two processes, copying is the one that primarily explains the distribution of traditions and traits throughout human populations.

In contrast, the reconstruction account argues that a learner’s goal is not to copy faithfully the behaviour of the model but instead to use pragmatic inferences, contextual cues, background knowledge, and other constructive processes in order to learn what they deem relevant in the behaviour and to adapt it to satisfy different goals in different contexts [6,7,12,13]. In contrast to copying, which is a content-neutral transmission mechanism (it does not matter what is being transmitted as everything is replicated in the same way), reconstruction is content-sensitive, as the content of information will affect the inferential processes [5,7,12,13,31,32]. These pragmatic inferential processes are argued to be the driving force of stability in cultural traditions, as people will tend to reconstruct information in similar ways due to shared heuristics.

Furthermore, learners will identify only those integral features that are relevant to them in a given context—other features of the to-be-produced action are then reconstructed inferentially. Reconstruction therefore predicts that, when a learner introduces variation, they do so non-randomly. The observed variation arises from convergent transformations—non-random modifications to inputs that reflect population-general biases in information processing—in line with content-sensitive reconstructive processes, as opposed to random copying errors [33]. Differences between a model and a learner’s productions that appear on incidental features are still considered irrelevant to cultural transmission under a reconstructive account, but differences on integral dimensions of a behaviour are driven by convergent transformations based on pragmatic inferences.

The article "Evaluating the relative contributions of copying and reconstruction processes in cultural transmission episodes" was published in 2021. Journal: PLoS One.

Distinguishing these two accounts empirically is difficult. Although they posit different underlying mechanisms, they predict similar patterns of behaviour with regard to the transmission of integral information features. Furthermore, different social learners may employ either or both mechanisms within the same transmission episode. For instance, some learners may copy while others reconstruct, or the same learners may even copy some features of a behaviour while reconstructing others. It is therefore important, when studying the population-level effects of cultural transmission, to know which individual cognitive mechanisms are responsible for which downstream effects on traditions.

One strategy is to use transmission chain experiments [34,35] and measure whether the information transmitted converges in some direction—reconstruction—or whether it transforms in a random manner—copying [36,37]. However, problems arise when transmitted information is highly stable across transmission episodes. While such stability may appear to reflect high-fidelity copying, this is not sufficient evidence against reconstruction, as a reconstructive process could well yield the same results if a model carried the same content that a learner would reconstruct. In such cases, reconstruction becomes indistinguishable from copying and leads to the same predictions: learners should reproduce the integral information features they observe and not reproduce more incidental features.

Given the fact that both processes can lead to superficially similar output forms, the key question is how can we evaluate the relative impact of copying and reconstruction on the transmission, transformation, and stabilisation of cultural traits? To do this, it is necessary to distinguish the relative impacts of copying and reconstruction processes within transmission episodes, and to identify what features of the behaviour are copied and which ones are reconstructed, and to what degree. An empirical approach that can distinguish between these two learning processes is therefore of paramount importance as it would shed light on the underlying cognitive mechanisms of social learning [12,38].

The article "Evaluating the relative contributions of copying and reconstruction processes in cultural transmission episodes" was published in 2021. Journal: PLoS One.

## Methodological approach

In order to distinguish between the processes of copying and reconstruction, we focus on a core prediction of the reconstruction account: that learners will adapt what they learn to fit their current task demands or context. By changing the production context between model and learner, therefore, it is possible to experimentally induce systematic deviations in the behaviours of both, and to predict the transformations that would be expected under both accounts. One way to introduce such deviations is to take advantage of incidental features of a behaviour that are embedded within integral information features.

Consider the tennis coach and student again. The novice can learn by observing his coach perform actions repeatedly, but the coach can in turn modify her behaviour to help scaffold her student’s learning. For example, when demonstrating a serve, she can slow down and exaggerate different parts of her movements in order to highlight hidden or non-obvious structures in the information. Exaggerations and intentionally slowing down are incidental action features in this case—they are not integral to serving a tennis ball, and not part of the to-be-learned information. However, these features are embedded within integral action features—swinging the racket in an overarm arc trajectory—which means it is not possible to simply omit them from a learner’s reproduction (the speed of the movement altogether, for example). Such embedded action features are common in teaching [39], coordination [40], and sensorimotor communication [41–43], and can result in changes to the dynamic profiles of movements in order to structure and communicate information.

By manipulating the context under which the model and learner produce behaviours such that the model introduces embedded action modifications while the learner need not, we can distinguish between predictions made by the two accounts. If learners are copying an input with embedded (but incidental) modifications, given that a learner cannot simply drop these modifications from their reproduction, they will replicate the actions they observe faithfully and introduce only random copying errors. As such, when the tennis novice comes to serve the ball he will slow down and exaggerate his movements in the same way as his coach. If learners are reconstructing, however, they should identify these modifications but, realising that they are incidental, will use pragmatic inference to reconstruct only the core, integral information. Under this account, the tennis novice will produce a tennis serve that is more similar to how the coach would serve a ball if they were actually serving in a tennis match.

The article "Evaluating the relative contributions of copying and reconstruction processes in cultural transmission episodes" was published in 2021. Journal: PLoS One.

The predictions of the two accounts are shown in Fig 1A–1C. A model has a private representation of some know-how around which her behaviour is distributed (Fig 1A). Her public behaviour may vary as a result of current context and situational constraints, but her core representation of the task remains stable. By manipulating the context using task instructions, we can introduce embedded modulations to the model’s actions that systematically deviate from this core representation, and use the resulting public display as input to a learner who does not share that context. When learners copy, any differences between their reproductions and the model’s public display that they observe will be due to random copying error. This will result in an internal representation of the information that is centred on the learned input and thus their reproductions will be more like the behaviour they have learned from (Fig 1B). On the other hand, when learners reconstruct then they will reproduce the behaviour in systematically transformed ways as they convergently transform the learned input back to their inferred understanding of the model’s internal representation. If they reconstruct the model’s representation successfully their own reproduction should look like what the model would have done had she not been instructed to embed action modulations (Fig 1C).

**Fig 1:** Predictions (A-C) of the copying and reconstruction account. A) A model’s behaviour follows a distribution (shown as normal for illustrative purposes only) centred on their representation of the to-be-transmitted information (Original; green line). By introducing deviation from this central representation through task instructions, the model produces a behaviour that falls away from the centre of this distribution (blue dot), which is passed on to the next generation (Learning; purple line). B) Under the copying account, participants will faithfully recreate what they see, introducing random copying errors. This will result in a distribution of behaviour (yellow) centred around the Learning action. C) Under the reconstruction account, participants will apply systematic transformations that converge back on the Original signal.

The primary goal of this paper is to present this methodological approach as a tool for evaluating the relative contribution of copying and reconstruction learning processes at play within episodes of cultural transmission. To do this, we apply our approach in a single-generation social learning episode involving the transmission of a complex behaviour that has multiple integral temporal and spatial dimensions. We explore in depth how information along these different integral dimensions is copied and reconstructed by introducing embedded context-driven action modifications.

The article "Evaluating the relative contributions of copying and reconstruction processes in cultural transmission episodes" was published in 2021. Journal: PLoS One.

The pedagogical context described above, where a model actively demonstrates their actions for a learner who understands the model’s pedagogical intention, is a good candidate for testing this approach, as a pedagogical intention to demonstrate behaviour should produce pedagogical cues that are embedded within task-integral action features such as the timing of the action (e.g. slowing down, exaggerating pauses, etc.). Pedagogical cues are behaviours that are intended to facilitate the transmission of information [44], and teachers show systematic and consistent strategies when modifying their actions suggesting the use of a general-purpose pedagogical repertoire that is presumed to be meaningfully interpretable by students [39].

The strength of this pedagogical context is that we can make clear predictions about both the nature of the pedagogical cues and how these will be interpreted. However, this context may also bias the learning context in favour of reconstruction—if a student recognises that a teacher is slowing down to be pedagogical, it may be easy to intuit that they are expected to produce the action at a faster speed. Although this is not a problem for a proof-of-concept, as our intention is to show that our approach is capable of empirically dissociating the copying and reconstruction accounts, it would also be useful to demonstrate the efficacy of this approach using a less clear-cut example. This is particularly relevant considering that the prevalence of teaching in real-world cultural transmission is disputed [44–47], and many studies of cultural transmission tend to focus on observational learning rather than didactic intentional transmission.

We also test our approach in a different social learning scenario where learners observe a model who is not demonstrating the action with a pedagogical intention but instead performing the action for aesthetic purposes. In this case, embedded incidental action features are not intended to be communicative or to facilitate the transmission of information. A learner who is watching a model perform the action to be aesthetic must therefore interpret what action features must be learned and what action features are intended to be stylistic without the support of intentional communication from the model. Applying our approach in this more challenging case allows us to show that it is possible to distinguish copying and reconstruction even in contexts that do not particularly favour one process over another.

We tested two learning conditions in an empirical validation study: one where the model demonstrated the action (Demonstration), and one where the model performed it for an audience (Performance). In both situations, at the beginning of the study learners were informed they would first see one of the model’s practice productions (i.e. where he produced the behaviour with no additional instructions), and when presented with the next video from the experimental condition, they were explicitly informed of the intention of the model that they learned from. This sequence of video presentations provided learners with a baseline behaviour to ensure that they would recognise performative or pedagogical signals embedded in the actions of the second video as intentional. We investigated how learners reproduced two integral features of the behaviour’s temporal dynamics—the absolute timing and the relative timing—with an aim to see whether participants copied or reconstructed either or both features.

The article "Evaluating the relative contributions of copying and reconstruction processes in cultural transmission episodes" was published in 2021. Journal: PLoS One.

## Empirical validation: A proof of concept

In order to characterise copying and reconstruction processes in an episode of observational social learning, we designed a single-generation transmission task using a short piece of music as the to-be-learned information. Music is an ecologically valid cultural item that can be transmitted and produced under different social and intentional contexts [48] and has been used successfully to study cultural transmission and evolution within the lab [49–51]. It is also a complex behaviour, comprising several dimensions that are integral to a production of the behaviour: the melody (the sequence of notes to play and the order in which to play them), and the timing, which may be decomposed to the absolute timing (the tempo at which to play the piece) and the relative timing (the rhythmic structure, or the proportional delays of particular inter-note intervals relative to each other).

For the purposes of the current study, we constrained the transmission of the melody such that participants could only progress with the study after learning the melody to a particular threshold (playing the specified notes in the correct order for ten consecutive trials). The two timing dimensions were allowed to vary, and these were the main variables of interest: temporal modulations of the piece, such as generally slowing down or speeding up (adapting the absolute timing), or exaggerating long or short pauses to allow for chunking of musical phrases (adapting the relative timing). Modulations along each of these timing dimensions can be incorporated into both performative and pedagogical productions. The empirical question, then, is whether learners who are exposed to these temporal modulations reproduce them in their own behaviour.

The article "Evaluating the relative contributions of copying and reconstruction processes in cultural transmission episodes" was published in 2021. Journal: PLoS One.

### Materials and methods

#### Participants

We recruited right-handed fluent English-speaking non-musicians who reported no history of neurological impairments or diagnoses, and normal or corrected-to-normal vision. We collected 16 participants to learn from each model seed, resulting in 32 participants in total (16M; 16F; M_age_ = 27y).

All experiments in this study were approved by the United Ethical Review Committee for Research in Psychology (EPKEB). Participants provided written consent before taking part in the experiment.

#### Apparatus

We used four Millenium MPS-400 Tom pads connected to a ddrum DDTi trigger interface to record responses, which participants produced with a wooden drum stick with a foam tip. Auditory feedback, metronome beats, and data recording was handled with a custom Max MSP patch that also recorded video and audio of the model and participants as they played the piece. Each drum produced a different MIDI tone, the pitch of which corresponded to a note from a pentatonic scale. Tones lasted for 250ms and the volume scaled to the force with which participants hit the drum.

Drums were positioned in front of the participant in a semi-circular arrangement. They were positioned on stands measuring 80cm high and 30cm apart (measured from centre to centre). Crucially, the drums were in the same position for the learners as for the model videos.

#### Stimuli

*Melody*. The melody that participants had to learn was constructed using four notes from a pentatonic scale (C,E,G,A) and consisted of 12 hits. The melody was designed such that a natural rhythmic structure emerged of chunking the first six notes into sets of three and the final six notes into pairs (i.e. 3-3-2-2-2). The reproduction of this rhythm (and its modulations) was the basis of our experimental investigation.

*Model videos*. Stimuli were collected by recording a musician (a male guitar player) using the same apparatus as participants used. The musician was instructed on the piece he was to play and was given a chance to practice it before playing it through in a further 30 videos (10 in each instruction context), from which three videos were selected for participants to learn from (one in each context). The three model example videos were selected after visually examining the inter-tap intervals (ITIs) and trajectories of these movements for obvious contextual modifications, as the ITIs were the measure of interest for the current study. Despite this selection, it is important to note that the model was not given any instructions as to *how* to modulate his actions to the given context: these were spontaneous modifications that he chose to make to the timing. The series of ITIs for each model sequence are shown in Fig 2A.

The article "Evaluating the relative contributions of copying and reconstruction processes in cultural transmission episodes" was published in 2021. Journal: PLoS One.

**Fig 2:** A. Inter-tap interval (ITI) sequences for each of the three model sequences. Interval index on the x-axis refers to the position of each ITI within the sequence (i.e. Interval index 2 refers to the interval between the first and second notes of the melody). B. Schematic timeline of the experiment. Participants start by watching the Original video through twice at the beginning of the experiment, without playing the piece back (green blocks). They then complete a turn-taking learning phase with the video (purple), where they watch the Learning video (the Performance or the Demonstration) and then play it back once each trial. For analysis purposes, this phase is split into two parts. Early learning trials (light purple) were used to gather data about errors and the number of trials taken to learn the piece. The last ten consecutive correct trials (practice trials; dark purple) were used as the criterion to end the learning phase and were used to derive data on the absolute and relative timings.

In the Original video context, the model played the piece under the instruction to practice it, and we take this sequence of ITIs to show what the expert model interpreted as the ‘pure’ rhythm (i.e. reflecting the model’s internal representation of the rhythm associated with this particular melody). One of these videos (repetition 7) was selected to be shown to participants as the Original, uninstructed production of the melody (ITIs shown in Fig 2A, left plot). The model’s Original productions were highly consistent across productions (mean cross-correlation: .97), indicating a stable representation that was not subject to a lot of natural variability.

In the Performance video context, the model was instructed to play the piece for an audience who would rate his performance in terms of style. This instruction created a performative context, which has an intentional component (to be stylish or aesthetic in a production), and a social component (the video will be watched by an audience). This led to lower consistency across productions (mean cross-correlation: .79), indicating the presence of variability in the model’s behaviour as a result of the instruction context. In the selected Performance, the model produced more extreme differences between long and short intervals relative to the Original, while maintaining a similar tempo to the Original (see Fig 1, middle plot). In operationalised terms, in this Performance the model introduced modulations to the relative timing of his actions but not to the absolute timing.

In the Demonstration video, the model was instructed to play the piece for somebody else to learn from watching him. This instruction created a pedagogical context, whereby the model intentionally introduced a series of modifications to the piece (e.g. slowing down and exaggerating the spatial and velocity profiles of his movements; [39]) that serve a social communicative goal: to scaffold information for the learner and facilitate learning. In this, as in the Performance video, there is an intentional component (to be pedagogical) and a social component (the video will be watched by a learner). As in the Performance context, this intentional context led to a lower consistency across productions relative to the Original productions (mean cross-correlation: .88), indicating context-driven variability when Demonstrating relative to the Original (practice) context, although to a lesser degree than when Performing. In the selected Demonstration video, the model produced exaggerations of long ITIs coupled with a general slowing down relative to the Original (see Fig 1, right plot). In operationalised terms, the model introduced modulations to both the relative timing of his actions and to the absolute timing.

The article "Evaluating the relative contributions of copying and reconstruction processes in cultural transmission episodes" was published in 2021. Journal: PLoS One.

The three videos that were selected to be shown to participants were edited to black out the top of the frame, obscuring all visual information about the model’s face and head movements. These videos, along with the timings of the 27 model productions that were not shown to participants, are available on the OSF project page.

#### Procedure

Participants came into the lab and completed the online Montreal Battery for the Evaluation of Amusia [52,53]. Participants were not excluded for low scores, but these scores (which evaluated participants’ sensitivity to modulations of scale, meter, and key) were collected for exploratory use.

Participants then sat at the experimental setup in front of the drum set. Participants were told that they would be learning to play a short piece of music on the drums in front of them. The experimenter played each note from lowest to highest (left to right, from the participant’s perspective) to show the mapping of the drums on the model’s video (the far left drum for the participant was on the right side of the screen).

The rest of the experiment timeline is shown in Fig 2B. Participants were told that they would first watch a video of a musician playing the piece they were about to learn so as to familiarise themselves with the task. To highlight the performative and pedagogical cues in the Learning videos, participants watched the Original video twice without playing it back. It is beyond the scope of the current study to see how such cues are interpreted without prior expectation to this Original practice context.

The article "Evaluating the relative contributions of copying and reconstruction processes in cultural transmission episodes" was published in 2021. Journal: PLoS One.

Then participants were told that they would now learn to play the piece by watching a different video of the same musician playing the same piece but under a different context. In **Learning from Performance** they were told that this musician had been asked to perform this piece for an audience, and that he knew that this video would be shown to people later on whose task would be to rate his performance in terms of style. In **Learning from Demonstration** they were told that the musician’s task was to demonstrate the piece for somebody else to learn, and he knew that his video would be later shown to people who would have to learn to play the piece from watching him.

Participants were told that they would watch the learning video (Performance or Demonstration) and then play back the musical piece that they heard. A trial was considered correct when the participant hit the prescribed drums in the prescribed order, and participants were explicitly told that this was the accuracy criterion. At no point were participants instructed to learn either the absolute or relative timing of the piece, and no mention was made of either ‘copying’ or ‘reconstructing’ the musical piece: participants were simply told to ‘play it back [after they heard it]’. Turn-taking with the model’s video continued until the participant had completed ten consecutive trials. These ten consecutive trials were termed the ‘practice’ trials, while all preceding trials (including any correct trials that were followed by an error trial) were treated as ‘learning’ trials.

During their production we recorded MIDI output, which we analysed, as well as video and audio recordings, which we did not analyse and do not discuss further. As this recording was started manually on each trial, participants were told that after they watched the video the experimenter would count them in (3-2-1) and then they would play the piece as best they could.

#### Design

There were two learning contexts: participants either learned by watching the selected model’s Performance or the Demonstration. This study was part of a larger study using motion-tracking where participants went on to perform and demonstrate the piece after the learning phase. For the purposes of the current study, only trials from the initial learning phase are reported.

For the purposes of validating our methodological approach, the key feature of the procedure was that all participants saw two videos: one Original video that was produced under the same instructions as participants themselves were given (to practice the sequence), and one Learning video that was produced under an intentional, social context, which the participants did not share and that introduced non-random modulations (embedded features) to an integral dimension of the information (rhythm). In order to analyse our data (see Data Analysis section) we investigated how learners reproduced two temporal features of the information: the absolute timing, measured by calculating the Euclidean proximity between the learned production and the model, and the relative timing, measured by calculating the structural similarity of participants’ ITI series to the model. Both of these metrics were calculated relative to the Original and to the Learning video, and the signed difference of these comparisons was treated as the dependent variable.

The article "Evaluating the relative contributions of copying and reconstruction processes in cultural transmission episodes" was published in 2021. Journal: PLoS One.

The two analyses, on two dependent variables, were computed as scores indicating evidence either in favour of reconstruction or copying, with a between-subjects factor of Learning context (Learning from Performance vs. Learning from Demonstration).

#### Data analysis

Data were collated from two stages in the learning process to address two principal questions (see Fig 2B). The first was whether participants found the melody easier to learn when the Learning video was a Performance or a Demonstration. To answer this question, sequence errors (failures to play the prescribed notes in the correct order) in early learning trials were tallied and compared. Fewer sequence errors in the Learning from Demonstration condition would indicate that participants found this seed easier to learn from than the Performance seed.

The second question related to how participants recreated the timings of the piece that the participants learned. To answer this question, only the final ten trials of the learning phase were analysed–the ten consecutive trials that participants had to play before the learning phase was considered complete. For each trial, we derived two values that compared the participant’s production against either the Learning video or the Original video: a measure of Euclidean distance, which indicated deviation in absolute timings, and a semi-partial correlation coefficient, which indicated structural similarity in the relative timings. The signed difference between these values (to the Original versus the Learning video) were used as directional evidence in favour of reconstruction (positive) or copying (negative).

*Learning rates*. Learning trials (all productions before the final ten consecutive correct practices) were kept separate from other data. We first investigated these learning trials to see if there were any differences in learning rate between the two learning conditions. The primary measures of learning rate were the number of trials required to reach the first of the ten practice trials (i.e., to learn the sequence) and the total number of error trials–because participants needed to complete ten consecutive practices, they could (and sometimes did) produce a run of correct videos and then make a mistake on a later trial. The total number of errors was collected to account for these late-learning errors. For example, a participant who only made a mistake on the first two learning trials would be considered as having completed 2 learning repetitions before the ten consecutive correct repetitions, with 2 erroneous repetitions. However, a participant who only made mistakes on their first learning trial and their tenth learning trial (after completing eight correct sequences) before going on to produce ten consecutive correct trials, would have completed 10 learning repetitions but made only 2 errors.

The article "Evaluating the relative contributions of copying and reconstruction processes in cultural transmission episodes" was published in 2021. Journal: PLoS One.

For all but two participants (due to a technical error), we collected scores on the online Montreal Battery for the Evaluation of Amusia (MBEA-O) on three dimensions: scale, metre, and key. High scores on this test indicate that participants struggled with the musical task, and this may be reflected in the learning rates.

*Data preparation*. The MIDI output from Max 7 included the drum ID, force, onset, and offset of each drum hit. There were ten of these for each participant, one per practice trial. The data were first checked for double taps where the drumstick bounced on the drum, registering as two taps when there was only one, and these were removed by deleting the intervening offset and onset. Inter-tap intervals (ITIs) were then calculated by subtracting the onset of a given note from the offset of the previous note. This generated a vector of eleven ITIs for each sequence that reflected the rhythmic structure of the piece (long ITIs reflect pausing at the end of rhythmic chunks).

Strings of ITIs were generated for each practice trial for each participant. These were compared against two of the three model videos (the Original video and whichever of the Performance and Demonstration videos participants had learned from watching, or the Learning video).

We analysed the ITIs of learners’ productions in two ways to examine how learners reproduced two temporal features of the melody: the first measure of interest was the *absolute* timing, defined as the numerical proximity of interval timings to the model’s productions, and the second was the *relative* timing, defined as the similarity of the internal rhythmic structure of the piece (i.e., the proportional relationship between ITIs).

*Absolute timing*. To examine the absolute timing, we calculated the Euclidean distance between ITI sequences using the root mean-squared difference (RMSD). This gives an approximate measure of proximity between productions in the potential production space. This measure of proximity is sensitive to the base tempo of the musical production, such that two productions with the same tempo would have a low RMSD, while productions with very different tempos will have a high RMSD. For each learner’s production, we calculated the RMSD proximity to the model’s sequence of interest (Original or Learning) and interpreted larger RMSD values as greater distance between the two compared productions.

The article "Evaluating the relative contributions of copying and reconstruction processes in cultural transmission episodes" was published in 2021. Journal: PLoS One.

RMSDs were calculated using Eq 1, where *x* is the ITI sequence of the learner’s production, *y* is the ITI sequence of the model’s production of interest (the Original or the Learning sequence), and *i* is the interval index (up to a maximum, *n*, of 11).


$$RMSD_{x}=\sqrt{\sum_{i=1}^{n=11}{\left(x_{i}-y_{i}\right)}^{2}}$$ (Eq 1)

In order to evaluate evidence in favour of copying or reconstruction, we calculated the signed difference between RMSD values for each learner’s production compared against the Learning and Original model separately. Difference scores were calculated as the RMSD to the Original model minus the RMSD to the Learning model, such that positive values indicate evidence for copying (smaller distance from the Learning video), while negative values indicate evidence for reconstruction (greater distance from the Learning video).

It is important to note that these proximity scores are sensitive to the RMSD between the models used. This is important because, as described above, the model slowed down the piece in the Demonstration but not in the Performance, resulting in a much larger RMSD relative to the Original for the Demonstration (RMSD = 840.03) than the Performance video (RMSD = 393.70). Given that the rationale of our approach is to see how participants copy or reconstruct exaggerated features of the signal, this difference in the model seeds means that this metric will be less sensitive to evidence one way or another in the Learning from Performance condition. However, this also means that the Learning from Performance condition will allow us to control for cross-generational differences in overall tempo (i.e. in the event that novice musicians produce generally slower melodies than the expert musician model): if we find greater proximity to the Demonstration video than the Original video in the Learning from Demonstration condition, this could be because participants are copying the absolute timing, or it could be because learners generally have a slower preferred tempo when playing the piece. In this case, we would expect raw RMSD values relative to the Learning video to be significantly larger in the Learning from Performance condition than in the Learning from Demonstration condition (as the Performance video was not slowed down, and would therefore be faster than the learners’ preferred tempo).

The article "Evaluating the relative contributions of copying and reconstruction processes in cultural transmission episodes" was published in 2021. Journal: PLoS One.

As such, we expect to find directional evidence (greater proximity to either the Original or Learning video) only in the Learning from Demonstration condition but not in the Learning from Performance condition. In the event that this evidence favours copying, we will then compare raw RMSD values to the Learning videos across conditions to see if this can be explained by a generally slower preferred tempo in learners (in which case we would expect to see significantly larger RMSD values to the Learning video when it is a Performance than when it is a Demonstration).

*Relative timing*. To examine the relative timing, we used semi-partial correlations (SPC), which examines the correlation among residuals in order to calculate the correlation of two variables holding a third constant. The two variables for each SPC coefficient were the participant’s production and the model’s sequence of interest (Original or Learning). The third constant was calculated using a grand average of all videos that the model made during stimulus generation minus the videos shown to participants. This grand average was used to control for the baseline similarity that one would expect to see between two ITI sequences of the same piece of music. SPC coefficients therefore show the residual relationship after controlling for the fact that they are two productions of the same melody, and greater SPC coefficient values indicate greater structural similarity between the two compared productions. The logic of this data analysis strategy is shown in Fig 3. Note that these coefficients are calculated only as a metric of similarity between two productions—rather than interpreting these coefficients on their own, we are interested specifically in comparing these metrics in relation to different model inputs.

**Fig 3:** Calculating similarity metrics for data analysis used four components: A) A grand average ITI sequence calculated across all videos produced by the model that were not shown to participants, across all three production contexts (n = 27 videos; Original, green; Performance, orange; Demonstration, blue). This model average (thick black line) served as a baseline of what sequence of ITIs would be expected of the model playing the piece in any given condition. B) Green. The ITI sequence of the Original video, which participants watched but never learned from. C) Purple. The ITI sequence of the Learning video (either the Performance or Demonstration). The ITIs of the Performance video are shown here for illustration. D) Red. The ITI sequence of the practice that participants made when learning from the Learning video (C). The centre of the Fig. shows how semi-partial correlations can be calculated between A, B, and D, or A, C, and D. The coefficients of interest that served as dependent variables (similarity metrics) are shown in bold, and show residual similarity of D (Participant practice, red) to either B (Original, green) or C (Learning, purple) while controlling for A (Model average, black).

The article "Evaluating the relative contributions of copying and reconstruction processes in cultural transmission episodes" was published in 2021. Journal: PLoS One.

In order to evaluate evidence in favour of copying or reconstruction, we calculated the signed difference between SPC coefficients for each learner’s production compared against the Learning and Original model separately. Difference scores were calculated as the SPC to the Learning model minus the SPC to the Original model, such that as with RMSD signed differences, positive values indicate evidence for copying, while negative values indicate evidence for reconstruction.

SPCs were calculated using the *spcor*.*test* function in the R package *ppcor* [54].

*Inferential statistics*. Signed difference proximity and similarity metrics were compared across conditions using linear mixed effect models. Models treated learning context (Learning from Performance vs. Learning from Demonstration) as a between-subjects factor, controlling for trial number (1–10 of the final learning trials), MBEA-O scores on the three subscales, and total number of learning trials. To model random effects, participant-specific intercepts and participant-specific slopes for trial number were calculated.

Total number of learning trials was included as a covariate in the mixed models analysis to control for greater exposure to the Learning video than the Original video, as the more times that a participant has seen the Learning video, the more that a copying mechanism may ultimately resemble the Learning input. It is important to note that this relationship is likely non-linear, as later exposures may be less influential than earlier exposures to the blended aggregate. The reported mixed models treat this effect as logarithmic, but it is worth noting that the same results are found when modelling a linear effect.

Mixed models were conducted using the *lmer* function in the *lmerTest* package in R [55,56].

### Results

#### Learning rates

Results of the learning rates are shown in Fig 4. Participants took generally fewer trials to learn from Demonstration (Fig 4; left) and made generally fewer errors when learning from Demonstration (Fig 4; right) than when learning from Performance. However, these differences were not significant (total trials: t(27.80) = -1.54, 95% CI [-8.59, 1.22], p = .135, d = -0.54; number of incorrect trials: t(27.72) = -1.34, 95% CI [-7.12, 1.50], p = .192, d = -0.47).

The article "Evaluating the relative contributions of copying and reconstruction processes in cultural transmission episodes" was published in 2021. Journal: PLoS One.

**Fig 4:** Boxplots showing learning rates when learning from Performance (orange) and Demonstration (blue). Learning rates calculated as total number of repetitions (left) and total number of errors (right). Points show individual participants.

One type of error that is worth noting was that, despite being shown the mapping of drums before learning, some participants nonetheless started to play back with the reversed mapping. Most realised their mistake and corrected themselves after one or two erroneous reproductions. Only one participant had to be explicitly instructed after 10 trials with the reversed mapping to reproduce the notes and not the positions of the sequence. Removing this participant did not affect the analysis of learning rate (total trials: t(27.55) = -1.71, 95% CI [-9.06, 0.82], p = .098, d = -0.61; number of incorrect trials: t(26.88) = -1.61, 95% CI [-7.61, 0.93], p = .120, d = -0.57), and they were retained for the full analysis.

Participants scores on the MBEA-O scales subscale did not correlate with number of learning repetitions (r = -.21; t(28) = -1.13, p = .270) or number of mistakes (r = -.18; t(28) = -0.99, p = .330). Neither did scores on the beats subscale (total trials: r = 0.26; t(28) = 1.43, p = .163; number of incorrect trials: r = .27; t(28) = 1.50, p = .146) or the keys subscale (total trials: r = -.05; t(28) = -0.24, p = .813; number of incorrect trials: r = .01; t(28) = 0.04, p = .972).

#### Absolute timings

The results of both the absolute timing proximity scores and the relative timing structural similarity scores are shown in Fig 5.

**Fig 5:** Raincloud plots showing the results of the proof-of-concept empirical study. Points show signed difference scores between proximity (top) and similarity (bottom) metrics of each learner’s reproduction relative to the Learning and Original seeds, such that positive values indicate support for a copying process while negative values indicate support for reconstruction. Results are shown separately for Learning from Performance (orange, left) and Learning from Demonstration conditions (blue, right). Boxplots and half-violin plots show the distribution of difference scores.

A mixed effect model of RMSD signed proximity scores found no effect of either the number of learning trials participants needed to learn the sequence (ß = -34.72, SE = 45.87, t(24.00) = -0.76, p = .457), or an effect of any of the MBEA-O subscale scores (ts<0.86). Similarly, there was no main effect of trial repetition number (ß = -0.67, SE = 6.48, t(29.00) = -0.10, p = .918), indicating that the tendency to copy or reconstruct the absolute timing did not systematically vary over time.

The article "Evaluating the relative contributions of copying and reconstruction processes in cultural transmission episodes" was published in 2021. Journal: PLoS One.

The model intercept was not significant, indicating that for participants in the Learning from Performance condition, there was no systematic bias towards copying or reconstructing the absolute timing (ß = -156.63, SE = 264.15, t(24.38) = -0.59,p = .559). Crucially, the model found a main effect of learning context (ß = 291.09, SE = 73.06, t(24.01) = 3.98, p < .001), where participants in the Learning from Demonstration context were significantly more likely to copy the absolute tempo than were those in the Learning from Performance context.

Given that the results of this analysis found evidence in favour of copying, we compared the raw RMSD values relative to the Learning video across the two learning conditions to see if this could be explained by participants having a generally slower preferred tempo than the model. To reiterate: if these results can be explained by the Demonstration video being produced at a slower tempo that matched participants’ preferred speed, then raw RMSD values should be significantly larger to the Learning video when it is a fast Performance than when it is a slow Demonstration. However, this did not appear to be the case, as RMSD values to the Learning video in the Learning from Performance condition (M = 673.51, SD = 341.15) were not significantly larger than in the Learning from Demonstration condition (M = 715.84, SD = 308.11; t(30) = -0.69, p = .493, d = -0.25). This indicates that, rather than learners simply having a generally slower tempo than the model, participants were copying the absolute timings of the melody in the video they learned from.

#### Relative timing

As with absolute timings, the mixed effects model of SPC signed difference scores found no effect of either the number of learning trials participants needed to learn the sequence (ß = 0.05, SE = 0.05, t(23.99) = 1.12, p = .276), or of trial repetition number (ß = 0.01, SE = 0.01, t(29.00) = 1.03, p = .312). There was an effect of one of the MBEA-O subscale scores: people who scored high on the scale subtest were more likely to copy the relative timing (ß = 0.89, SE = 0.40, t(24.01) = 2.22, p = .036), but this was not true for the keys subtest timing (ß = -0.17, SE = 0.34, t(23.99) = -0.49, p = .632) or, importantly, the beats subtest, which was the only test relating to musical sensitivity to timing (ß = -0.38, SE = 0.27, t(24.00) = -1.40, p = .174).

For relative timing, the mixed model did find a significant negative intercept (ß = -0.58, SE = 0.26, t(24.42) = -2.19, p = .038), indicating that participants in the Learning from Performance condition were significantly more likely to reconstruct than to copy the relative timing of the melody. This bias was numerically stronger, but not significantly different, in the Learning from Demonstration condition (ß = -0.03, SE = 0.07, t(24.00) = -0.41, p = .684), indicating that participants did not differ across learning contexts in their tendency to reconstruct the relative timing of the piece. These results of the analysis of SPC structural similarity measures indicate that, in both learning conditions, participants reconstruct the rhythm of the model’s Original production, away from the sequence they learned from watching.

The article "Evaluating the relative contributions of copying and reconstruction processes in cultural transmission episodes" was published in 2021. Journal: PLoS One.

## Discussion

### Empirical proof of concept

We present an experimental proof-of-concept using our proposed methodological approach for the study of cultural transmission to distinguish between copying and reconstruction processes within a single-generation transmission episode. We find that when varying the task context between a model and a learner in such a way that the model introduces embedded incidental modifications to their actions, learners show evidence of using both copying and reconstruction processes in their own reproductions. Specifically, learners’ reproductions of the absolute timing were better described by a copying mechanism than a reconstruction mechanism: Their productions are closer to the video they learn from than to the original, unmodulated production of the model. On the other hand, learners’ reproductions of the relative timing were better described by a reconstruction mechanism than a copying mechanism, as the series of ITIs are more similar to the model’s original, unmodulated production than to the video they learned from watching. It is worth noting that the distribution of values in SPC scores in participants who learned from watching a Demonstration appears to be somewhat bimodal. This suggests that the tendency to copy or reconstruct may be sensitive to individual differences within a population; a relationship which merits future study.

A point to note about the analysis of SPCs is that, because these are compared against different productions while controlling for a grand average of 27 unseen videos, they may be sensitive to differences in these videos unrelated to learning. Indeed, these stimuli were created to test the idea that non-random variation in a production aimed at satisfying a local task-relevant intention (performative or pedagogical) would lead to particular deviations from the ‘norm’ Original behaviour. As is evident from Fig 2A, this was successful as Performance and Demonstration contexts led to different patterns of ITIs from the Original. However, if these productions are outliers in the potential space of timings that the model might produce, and if they are very different to the other productions that make up the grand average used in SPCs, this could affect the strength of residual correlations after controlling for the grand average of the model’s other productions. To explore whether this was the case, we compared the three model videos of interest against the grand average with simple correlations. The Performance video had a lower correlation with the grand average in terms of timings (r = .87) than the Original video (r = .94), suggesting that the Performance video could have been considered particularly idiosyncratic. However, the model’s Demonstration video did not have a lower correlation with the grand average (r = .95) than the Original, suggesting that the evidence for reconstruction seen here cannot be explained by this difference in the seeds.

The article "Evaluating the relative contributions of copying and reconstruction processes in cultural transmission episodes" was published in 2021. Journal: PLoS One.

The initial presentation of the Original video to participants at the beginning of the experiment, which was intended to highlight the presence of performative or pedagogical cues, posed a potential confound. While this initial exposure provides reconstruction with a template to work back to, it also provides an additional input to copying mechanisms that may have prompted either a selection pressure for the Original (biased copying [10,57]) or led to a blended copying approach where the Original and the Learning video inputs were combined into a weighted aggregate [19]. In either case, the presentation of another input could have biased participants to copy the Original in some way, resulting in a deviation from the Learning input that would be indistinguishable from reconstruction. We did not anticipate this as a confound, as participants did not physically practice the melody when observing the Original video—and, when participants did start to practice, none of them played it through correctly the first time, indicating they were not holding it in memory with enough fidelity to copy it. However, it is prudent to control for such eventualities, to rule out a more indirect form of copying. In either case, the premise would be that, having seen the Original video at the beginning, participants would remember the timings of that video well enough to copy it (either directly, or blended with the input from the Learning video). In such a case, greater similarity to the Original video should decrease the more trials participants took to learn the sequence: if participants were demonstrating biased copying for the Original, then this should only be seen for participants who held the video in memory well enough to learn the sequence relatively quickly, whereas if they were blending the inputs in a weighted aggregate then the similarity to the Original should decrease as exposure to the Learning video increases. On the other hand, neither unbiased copying without blending nor reconstruction would predict any effect of the number of learning trials on outcome similarity on any measure. Our analysis including number of learning trials as a covariate found no effect on any outcome, indicating that our results were unlikely to be explained by biased or blended copying.

The article "Evaluating the relative contributions of copying and reconstruction processes in cultural transmission episodes" was published in 2021. Journal: PLoS One.

The current study introduces several key methodological changes from established transmission chain paradigms. In transmission chain studies, participants usually contribute only a single production: they observe the model and then their single attempt to reproduce the behaviour is used as a seed for the next generation. In contrast, we allowed both learners and the model to practice the behaviour and presented non-practice examples from the model that were produced under different contexts. This allows us to identify factors affecting the transmission of information independently of participants’ experience (or lack thereof) with the task—our results cannot be explained by participants simply becoming familiar with the behaviour as we ensured that all participants gained a degree of proficiency in the task [35]. By showing that it is possible to approximate a degree of proficiency in the lab while still observing cross-generational change, we ensure that emergent variations are due to the evolution of information through transmission rather than the result of uncertainty in one-shot early learning.

The experimental criterion of ten consecutive correct practices ensured faithful copying of one integral dimension—the sequence of notes—while allowing others—the absolute and relative timing, in which context-driven modifications were embedded—to vary freely. In contrast, transmission chain experiments typically measure only a single variable or dimension when evaluating the fidelity of transmission [35]. Furthermore, when analysing the dimensions of interest, we also differentiate between integral and embedded incidental features and focus on the expression of these embedded features. Given that tasks and metrics in cultural transmission studies are often simplified to reduce the degrees of freedom along which reproductions can vary, an approach that exploits the natural complexity in ecologically valid complex actions can offer unique and compelling insights into the underlying learning processes that govern cultural transmission.

The article "Evaluating the relative contributions of copying and reconstruction processes in cultural transmission episodes" was published in 2021. Journal: PLoS One.

Our empirical proof-of-concept study indicates that both copying and reconstruction can play a role in observational social learning and show that, using this approach, it is possible to disentangle the social learning processes that subserve the acquisition of relevant features of a complex transmitted behaviour.

### General discussion

The aim of this study is to provide a tool for future work that can differentiate copying and reconstruction processes in particular learning episodes. Copying and reconstruction posit different cognitive mechanisms for social learning, and these mechanisms have consequences when scaling back up to the transmission and stabilisation of cultural traditions across generations. With complex behaviours that encompass a range of different features that must be learned and expressed upon reproduction, the social learning mechanisms at work could therefore directly impact the flexibility and rigidity of cultural traits at the population level. The approach that we present offers an opportunity for future work examining the role of individual cognitive mechanisms in cultural transmission and cultural evolution. The core of our approach can serve as a useful new tool when designing transmission studies that exploit changes in task context to examine mechanisms of social learning.

Our approach also raises questions that are relevant to the study of both cultural evolution and social interactions, about the mechanisms by which learners identify and interpret contextual cues in order to understand transmitted information. For example, although there is a well-established literature showing that observers can use action kinematics to decode both instrumental [58–61] and communicative intentions [39,62,63], it remains an open question whether people can recognise these embedded signals spontaneously, and whether the same embedded signals can be interpreted differently merely by manipulating task instructions. To what extent these contextual signals rely on pragmatic common ground assumptions, and how these assumptions impact what learners copy or reconstruct, remains an interesting avenue for empirical research.

We outline an innovative methodological approach to studying transmission episodes that can make competing predictions about copying and reconstruction by exploiting incidental action modulations that are embedded in integral dimensions of the behaviour. The key elements of our approach are as follows: learners should learn from a seed that was produced under a context they do not currently share, with this context having elicited embedded contextual modulations of the to-be-learned behaviour in the model, and the behavioural output of learners’ productions should not just be compared to their input, but to other instances of the model’s behaviour *across different production contexts*. We present a proof-of-concept using music as a candidate behaviour and temporal exaggerations as the embedded incidental information, but this approach is generalisable to a range of cultural phenomena.

The article "Evaluating the relative contributions of copying and reconstruction processes in cultural transmission episodes" was published in 2021. Journal: PLoS One.

For example, this approach could be used to explore how learners acquire flexible motor skills that involve adapting to physical situational constraints, such as stone knapping, pottery, or textiles. Such skills involve variability in material and environmental properties that are associated with compensatory motor adaptations [64]. Understanding what learners copy and what they reconstruct from observations of models acting under different physical constraints can offer some insight into how learners extract stable regularities about flexible skill sets through observation.

This methodology can also be extended beyond the motor domain and apply to the study of artefacts themselves. Transmission chain studies frequently use tasks involving some technical engineering (e.g. building a tower out of spaghetti, or constructing a paper aeroplane). While these are likely too simple to adapt to the current approach, as previous experience with these tasks can lead to a ceiling effect in transmission fidelity, tasks using more complex artefacts, e.g. [65], that can be analysed with more fine-grained morphological analytic approaches [66,67] may offer enough meaningful variation across contexts to benefit from our methodology. This could allow future researchers to identify what morphological features learners copy and what they reconstruct across different production contexts, such as: pedagogical vs. non-pedagogical contexts, collaborative contexts where artefacts must be passed along to another person to be completed vs. contexts where the full production pipeline is completed by the same person, or contexts where different intentions are prioritised during the manufacturing process such as speed or accuracy. Scaling up from the level of a single production, studying the transmission of artefacts through a transmission chain with the knowledge of what features participants are copying or reconstructing would allow researchers to make specific predictions about the propagation and stability of these features over the course of successive generations [35].

Contextual modifications and transmission chains do not apply only to techniques or actions. A popular paradigm in transmission chain studies involves using verbal communication of narratives, in the style of the children’s game Telephone [36,68]. Narration and storytelling are also cases where narrators can and do make contextual modulations in order to satisfy particular intentions such as to be interesting or convincing [69]. As in the current study, such modulations may involve embedded timing modulations affecting the prosody of the speech (such as when producing particularly emotive or evocative speech), but these can also apply to other linguistic devices that can be identified and studied using discourse analytic approaches [70]. Understanding how listeners or learners respond to motivated storytelling from biased sources is an important question with a growing body of literature [71–75], and examining this in a cultural transmission context to see how and what receivers copy and reconstruct from narratives (and conversely, whether and how narrators can anticipate what details will be copied and reconstructed) could offer useful insights.

The article "Evaluating the relative contributions of copying and reconstruction processes in cultural transmission episodes" was published in 2021. Journal: PLoS One.

Our current empirical study indicates that both, copying and reconstruction processes, are at play in social learning episodes, and that this methodological approach can be used to distinguish them by their relative effects on the outcome of a social learning episode. This is a valuable tool for the study of cultural transmission, as this can allow researchers to draw links between cultural phenomena and individual psychological learning mechanisms, as well as to identify what local contextual factors affect the expression of different learning mechanisms. For example, in the case of the tennis novice who observes his teacher’s exaggerated dynamics, we might expect reconstruction given that the learner likely has a pre-existing representation of what a tennis serve should look like from watching the sport, and so the goal of a demonstration is to provide scaffolding that helps correct or shape this pre-existing representation in ways that can be readily reconstructed without having to adopt the same scaffolding behaviours. On the other hand, in cases where the difference between incidental and integral features is more opaque, due to a lack of experience, or where the risks of incorrectly dismissing integral features outweigh the costs of reproducing incidental action features, it is very plausible that learners would be more likely to faithfully copy. When these learners go on to produce and develop these behaviours, the mechanisms they used to initially acquire the behaviour may affect how later information is shaped, stored, and integrated. Crucially, the methodological approach that we propose can distinguish these processes in different transmission episodes and across different types of phenomena and is impartial in that it makes clear and testable predictions about both copying and reconstruction.
